# Image Reconstruction Based on Progressive Multistage Distillation Convolution Neural Network

**DOI:** 10.1155/2022/9637460

**Published:** 2022-05-09

**Authors:** Yuxi Cai, Guxue Gao, Zhenhong Jia, Liejun Wang, Huicheng Lai

**Affiliations:** College of Information Science and Engineering, Xinjiang University, Urumqi 830046, China

## Abstract

To address the problem that some current algorithms suffer from the loss of some important features due to rough feature distillation and the loss of key information in some channels due to compressed channel attention in the network, we propose a progressive multistage distillation network that gradually refines the features in stages to obtain the maximum amount of key feature information in them. In addition, to maximize the network performance, we propose a weight-sharing information lossless attention block to enhance the channel characteristics through a weight-sharing auxiliary path and, at the same time, use convolution layers to model the interchannel dependencies without compression, effectively avoiding the previous problem of information loss in channel attention. Extensive experiments on several benchmark data sets show that the algorithm in this paper achieves a good balance between network performance, the number of parameters, and computational complexity and achieves highly competitive performance in both objective metrics and subjective vision, which indicates the advantages of this paper's algorithm for image reconstruction. It can be seen that this gradual feature distillation from coarse to fine is effective in improving network performance. Our code is available at the following link: https://github.com/Cai631/PMDN.

## 1. Introduction

Single image super-resolution reconstruction (SISR) is one of the classical research problems in the field of computer bottom vision. It aims to recover the corresponding high-resolution (HR) image from the degraded low-resolution (LR) image by using certain technical means. SISR is an inherently ill-posed problem because there are a large number of high-resolution images in the real world that are degraded in very different ways to obtain similar low-resolution images [1].

In recent years, benefiting from the rapid development of deep learning, it has been shining in the field of computer vision, such as target tracking [2–4], blind image quality evaluation [5–10], and face processing [11, 12]. Currently, a large number of deep learning-based SISR algorithms have emerged and have achieved better results than traditional algorithms in both objective metrics and subjective vision.

Dong et al. [13] first applied deep learning to the field of image restoration in 2014, proposed a shallow convolution neural network with three convolution layers, and established the direct mapping relationship between LR image and HR image. Subsequently, researchers began to use deep learning technology to construct deeper convolution neural networks, such as [14–19], which have achieved better performance than SRCNN. However, with the increase in network depth and width, the performance is significantly improved, but the network becomes difficult to converge. In order to solve the problem that the network is difficult to domesticate, Kim et al. [20] proposed residual learning for the first time to solve the problem that the gradient disappears due to the increase of network depth. Subsequently, Zhang et al. [21] constructed a very deep dense connection network by using the residual connection. The network makes full use of the hierarchical features of LR images to improve the network's performance but also causes the redundancy of a large amount of information to a certain extent. Due to the difference in scale, aspect ratio, and convolution stage, the same or similar objects will behave differently in the image. The information can be well captured by various levels of features, which will help to obtain good reconstructed images. Tai et al. [22] performed the exchange of feature information by using long and short jump connections in MemNet networks as a way to exploit the hierarchical features at different stages. However, in the memory block, the current convolution layer cannot directly access all convolution layers in the subsequent block and thus cannot fully utilize the local feature information, which limits the capability of long and short jump connections. Zhang et al. [23] proposed the information continuity mechanism, which enables each convolution layer in the current block to directly access the output information of the previous block through a dense connection so as to realize the continuous transmission of information. With this information continuity mechanism, the network makes full use of the hierarchical features and obtains good reconstruction results, but it also results in redundancy of hierarchical information and a huge computational overhead. The distillation mechanism was then introduced into SISR, which distills some fine features from many similar features and solves the problem of information redundancy in feature fusion. In the case of limited network size and computation, IDN [24], IMDN [25], RFDN [26], etc. allow the network to achieve good reconstruction performance through the distillation mechanism.

IMDN and RFDN both distill one-fourth of distilled features from total input features with the help of the distillation mechanism and then further process output features of the previous base block by convolution layers. In this way, the network explicitly acquires the fine-grained features in each layer. We believe that each distillation operation distills only a quarter of the total input features, and this rough one-step distillation method will omit many critical features, which may play an important role in improving the network performance. Secondly, the small base blocks of IMDN and RFDN only process output features of the previous small base block and distill a small portion of the features from it. This feature processing way will make the network feel the previous redundant feature information again and increase the burden of the network. Finally, many reconstruction algorithms use the operation sequence of channel compression and recovery in their proposed channel attention to model the relationship between channels. We believe that after channel compression, channel recovery is carried out through the convolution layer, which is difficult to restore the channel information state before compression. In other words, compressing and then recovering this channel operation way will cause the loss of some channel information.

In order to solve the problem of the loss of some important features caused by rough feature distillation and the loss of key information in some channels caused by the compressed channel attention in the network, we propose a progressive multistage distillation network, and the important features are distilled step by step from coarse to fine. To maximize the performance of the network, we propose weight-sharing information lossless attention block, which effectively avoids the loss of channel information and enhances the channel characteristics with the help of the auxiliary branch of weight sharing, allowing the network to extract the key information in different channels. For this paper, the main contributions are as follows:

1. The weight-sharing information lossless attention block (WSILB) is proposed. It models interchannel dependencies uncompressed by 1 × 1 convolution layers and enhances channel characteristics by weight-sharing auxiliary branches, effectively solving the problem of channel information loss due to channel compression, at the same time, allowing the network to focus on critical channel information more precisely.
2. Dual branch information calibration reservation block (DCRB) and progressive multistage distillation block (PMDB) are designed. WSILB is integrated into DCRB, which can adjust the channel feature response adaptively and retain the underlying feature information through another branch. On the other hand, PMDB distills fine features from the input features step by step, retaining the corresponding important features of each stage, greatly reducing the problem of loss of key features in rough distillation, and enhancing the ability of the network to learn and represent key features.
3. A progressive multistage distillation network (PMDN) is constructed. In the reconstruction phase, it introduces WSILB into it, and through the step-by-step up-sampling strategy, the network has enough high-frequency information to use. In particular, we combine the step-by-step sampling strategy with the weight-sharing strategy to work together in the reconstruction phase. Importantly, PMDN produces competitive reconstruction results and achieves a good balance between network performance, number of parameters, and computational complexity.

## 2. Related Work

The hierarchical features of different stages contain different feature information, and the information has varying degrees of contribution to improve the performance of the network. How to effectively aggregate the hierarchical features of different stages while keeping the network lightweight is also a problem that researchers have been thinking about.

In order to integrate the hierarchical features of different stages as much as possible, Li et al. [27] designed a multiscale residual network, which combines the image features obtained by local multiscale feature blocks with global features to maximize the use of image features in LR space. Subsequently, Wang et al. [24] introduced the idea of distillation in IDN, where the features processed by the convolution layer are divided into two parts after the channel splitting operation, a part of the features continues to be deepened by the convolution layer, and the remaining features are stitched together with the original input features and jump transferred to the end of the enhancement block for the spanning fusion of different local features in order to strengthen the network learning of LR contour region. Inspired by Wang, Hui et al. [25] proposed a multidistillation network, which retains some of the intermediate features while further dealing with the remaining features. With this channel splitting approach, the network can aggregate feature information at different levels, and thus, the network performance is improved. Jiang et al. [16] use dense hierarchical connections in networks to fuse information about hierarchical features at different stages. Yi et al. [17] merged multiscale structure and hybrid convolution into the network to capture the dependencies of features at each stage. Liu et al. [26] designed a residual distillation network, which uses 1 × 1 convolution layers instead of channel splitting operation for information distillation; this operation injects some flexibility into the network, and the network performance is further improved. However, the refinement of features using 3 × 3 convolution layers with residuals cannot extract diverse feature information. In addition, it cannot guide the network to focus on the key feature information so that it cannot provide sufficiently rich local high-frequency information for the final recovery of the image.

LR images have rich low-frequency information, but we pay more attention to the high-frequency information which is conducive to image detail recovery and how to effectively bypass the low-frequency information and extract the richer high-frequency information, which also needs our consideration. The existing channel attention mechanism [28] explicitly models the interdependence between feature channels, in which the average pooling operation also effectively improves the objective index, but it lacks the description of image texture and edge information, resulting in a certain degree of smoothing and blurring in the reconstructed image. To address this problem, Hui et al. [25] designed a contrast-aware channel attention block by using standard deviation and average value instead of global average pooling in the channel attention block, which effectively recovered the edge texture details of the reconstructed image. However, the module spends some attention to focus on complex low-frequency information, resulting in a partial waste of resources. Zhang et al. [29] designed a deep residual channel attention module that adaptively readjusts the features of each channel by modeling the interdependence between feature channels, while allowing rich low-frequency information to spread directly through multiple jump connections, making the network more focused on the learning of high-frequency information so as to achieve a good recovery effect. Liu et al. [30] use convolution and pooling layers to further enhance the perceptual field of spatial attention so that the network can learn more contextual information. In addition, Wang et al. [31] proposed recurrent residual channel attention block, which further improves network performance by introducing circular connection in the attention block while keeping the parameter constant.

## 3. Our Algorithm

In this part, we first introduce the progressive multistage distillation network proposed in this paper and then introduce the important components of the network in detail.

### 3.1. Overall Framework

As shown in Figure 1, the progressive multistage distillation network (PMDN) consists of shallow feature extraction block, progressive multistage distillation block, and reconstruction block. In this paper, *I*_LR_ and *I*_SR_ are represented as the input and output images of the network, respectively. According to the research of [32, 33], we only use a 3 × 3 convolution layer to extract the shallow features I_LR_:

(1) $$\begin{array}{c} F_{0}=Conv_{3\times 3}\left(I_{LR}\right), \end{array}$$

where Conv_3×3_(.) represents the convolution operation with a convolution kernel of 3 × 3 and *F*_0_ represents the shallow features extracted by the convolution layer. Then, *F*_0_ is used as the input of progressive multistage distillation block to deepen the feature in order to learn more discriminating feature representation.

Assuming that there are *d* progressive multistage distillation blocks (PMDB), the output features *F*_*d*_ of *d*th PMDB are expressed as

(2) $$\begin{array}{c} F_{d}=H_{\text{PMDB},d}\left(F_{d-1}\right)=H_{\text{PMDB},d}\left(H_{\text{PMDB},d-1}\left(\ldots \left(H_{\text{PMDB},1}\left(F_{0}\right)\right)\ldots \right)\right), \end{array}$$

where *H*_PMDB,*d*_(.) denotes the *d*th PMDB with composite function. *F*_*d*_ denotes the local fusion features extracted after the *d*th PMDB processing, and more details about PMDB will be detailed in Section 3.3.

After multiple PMDB processing, the discriminating features we have learned are fed into the reconstruction block with attention and then restored to the corresponding target size. The operation process is expressed as follows:

(3) $$\begin{array}{c} F_{n}=H_{U-\text{WSILB}}^{n}\left(H_{U-\text{WSILB}}^{n-1}\left(\cdots H_{U-\text{WSILB}}^{0}\left(F_{d}\right)\cdots \right)\right), \end{array}$$

where *H*_*U*−WSILB_^*n*^ represents the *n*th U-WSILB block, *F*_*n*_ represents the output features of the *n*th U-WSILB, and more information about U-WSILB will be described in Section 3.4.

To compensate for the problem of losing some of the underlying information in the continuous deepening process of the features, we use the traditional interpolation algorithm to up-sample *I*_LR_ to the corresponding size and then supplement the information with a jump connection to generate the final *I*_*SR*_:

(4) $$\begin{array}{c} I_{SR}={\text{Conv}}_{3\times 3}\left(F_{n}\right)+H_{\text{up}}\left(I_{\text{LR}}\right). \end{array}$$

Here,  *H*_up_(.) denotes the bilinear interpolation up-sampling operation.

Based on previous research work, we use *L*_1_ loss function for the optimization of network parameters. Given a training set {*I*_*LR*_^*j*^ ,*I*_*HR*_^*j*^}_*j*=1_^*j*=*N*^ containing many image pairs, where N represents the number of training image pairs, and the loss function with parameters used in this paper is expressed as

(5) $$\begin{array}{c} L\left(\theta \right)=\frac{1}{N}\sum_{1}^{N}{\left\|H_{\text{PMDN}}\left(|I_{LR}^{j}\right)-I_{HR}^{j}\right\|}_{1}. \end{array}$$

Here, *θ* denotes the network parameters to be optimized and *H*_PMDN_(.) represents the progressive multistage distillation network.

### 3.2. Weight-Sharing Information Lossless Attention Block (WSILB)

Most of the channel attention use global average pooling to represent the channel characteristics, but the average value is difficult to fully represent the feature information in the channel, which leads to the poor reconstruction effect to some extent. Secondly, these channel attention use the way of channel compression and recovery to model the relationship between channels, which will lose part of the channel information in varying degrees. Different from the previous types of channel attention, we design a weight-sharing attention block with lossless channel information as shown in Figure 2.

We use the sum of standard deviation and average of channel information to characterize the channel properties. To enhance the network's attention to detailed information such as edge textures, we construct weight-sharing auxiliary branch using a maximum pooling operation for enhancing the channel properties. In order to lighten the module as much as possible, we directly model the interrelationships between channels using 1 × 1 convolution layers in an uncompressed fashion, avoiding the previous problem of information loss due to channel compression. In addition, the two branches use the same convolution weight, which keeps the channel properties in the same mapping relationship. Then, we sum the outputs of the two branches to generate attention mask by the sigmoid function.

### 3.3. Progressive Multistage Distillation Block (PMDB)

To avoid the previous crude feature distillation approach as well as to retain more important feature information, we designed a progressive multistage distillation block that allows the network to learn a more discriminating feature representation through progressive feature compression, and the internal structure of the block is shown in Figure 3a.

Unlike IMDN, RFDN, and other distillation methods that distill small parts of features from input features in a coarse manner, we gradually distill some key features from input features from coarse to fine. We distill features from distillation features stage by stage.

The progressive multistage distillation block (PMDB) consists of dual branch information calibration reservation block (DCRB), convolution layer, and WSILB, where the internal structure of DCRB is shown in Figure 3b.

For the DCRB, we use 1 × 1 convolution layer for feature compression to reduce the redundant feature information and alleviate the amount of network computation. Immediately after that, we use the convolution layers of different convolution kernels to deal with the same features in parallel so as to realize the feature fusion under the multisensory field. At the same time, we use attention blocks to enhance the network learning of key features. Reference [34] argues that channel attention may discard some relevant details of features that would be difficult to regain at deeper network levels. Therefore, we open a second branch that processes the features using 3 × 3 convolution layers to preserve the underlying information in the features. Finally, we concatenate the output features of two branches together according to the channel dimension and use the 3 × 3 convolution layer to establish channel dependencies at a distance and then distinguish the importance between channels with the help of WSILB.

For PMDB, one of the important components of the network, we gradually distill the relatively critical features in each stage from coarse to fine. Specifically, we first use DCRB to process the input features and then use 1 × 1 convolution layer to distill the features, with the distillation rate set to half of the original total features. We will continue to learn the deep feature relationship from the distillation features of the previous stage through DCRB and then use the convolution layer to select the relatively important features in this stage. By analogy, the network gradually distills out the important features of each stage; meanwhile, the receptive field of the network is also expanded. With this progressive stage-by-stage distillation way, the network learns the distillation feature representation of each stage from coarse to fine, and the depth of the network is further deepened. Finally, we splice the distillation features of each stage together, which is different from the previous stage feature fusion, we abandon the 1 × 1 aggregation layer and directly use the 3 × 3 convolution layer to establish a large-scale feature fusion relationship, and then use the WSILB to enhance the network's extraction of key information in the fusion features so that the network can learn more powerful feature representation. In addition, we use residual connections at the end of PMDB to perform jump propagation of the original information in order to benefit from residual learning and to speed up the backpropagation of gradients in network optimization.

### 3.4. U-WSILB

In some previous reconstruction algorithms, the reconstruction block of the network is usually composed of convolution layer and subpixel convolution layer [35], and the attention mechanism is rarely introduced into the reconstruction process, resulting in the key features difficult to play their due role. On the other hand, for large-scale reconstruction tasks, such as ×4, if there is not enough high-frequency information, it is difficult for the network to achieve satisfactory reconstruction results. Aiming at the above two points, we construct U-WSILB, whose internal structure is shown in Figure 1, which is composed of the nearest neighbor interpolation algorithm, WSILB, and two convolution layers. The NNIA in Figure 1 represents the nearest neighbor interpolation algorithm.

In U-WSILB, we abandon the subpixel convolution and use the nearest neighbor interpolation algorithm to achieve the up-sampling operation, mainly because the subpixel convolution layer brings a large number of parameters to the network but also cannot achieve the corresponding recovery effect. In this paper, we use the convolution layer to further establish the correlation between channels for the interpolated features. In order to distinguish the importance between channels and play the role of some key features, we use WSILB to enhance the network's attention for key channels to achieve the purpose of improving network performance.

In order to cope with the large-scale reconstruction task, the network still has enough available high-frequency information while ensuring that each step of the up-sampling is optimal; we use the distributed strategy to carry out step-by-step up-sampling until the target size is reached, such as the ×4 reconstruction task, we divide it into two cascaded ×2 reconstruction tasks, and we use the weight-sharing strategy to further reduce the number of network parameters.

## 4. Experiment and Analysis

We trained the network using DIV2K, a high-quality data set containing 1000 images published by Timofte et al. [36], and the Flickr2K data sets containing 2650 images. For testing, we used four standard benchmark data sets, Set5, Set14, B100, and Urban100, and used the objective indexes of peak signal-to-noise ratio (PSNR) and structural similarity index measure (SSIM) [37] to quantitatively analyze the reconstruction results and convert the image from RGB color space to YCbCr color space. Only Y channels are trained and tested.

### 4.1. Experimental Environment and Parameter Settings

In this paper, 24 image patches of size 192 × 192 are randomly selected as the input of the network in the ×2, ×3, and ×4 reconstruction tasks. 1000 backpropagation iterations constitute 1 epoch with an initial learning rate of 0.0002, and the learning rate decays to half of the original after every 200 epochs. The network uses 6 PMDB, the slope of Leaky-Relu is set to 0.05 in the negative range, and the Adam algorithm is used to optimize the network gradient. The algorithm in this paper is built under the PyTorch deep learning framework, the experimental hardware platform is NVIDIA Tesla V100-PCIE-16 GB, and the software environment is Windows 10 operating system.

### 4.2. Ablation Experiments

In order to verify the effectiveness of the network design, we conducted ablation experiments on some important blocks. All the ablation experiments are built on ×4 reconstruction task, and the results are obtained by training 400 epochs, which can better test the effectiveness of each block design in the network.

*Verifying the rationality of the WSILB design*: first, we gave four design schemes as shown in Figure 4. Type A is the scheme we used in the article. Unlike type *A*, type *B* uses two convolution layers to establish the dependencies between channels separately, that is, the features of the two branches do not have the same mapping relationship. Type C uses the sum of standard deviation, average, and maximum to characterize the channel properties. Type *D* directly uses the sum of standard deviation and average to characterize the channel properties. All types of attention blocks deal with the feature channel without compression. We use *B*, *C*, and *D* types of attention blocks instead of A type of attention blocks for experimental verification, and the experimental results are shown in Table 1.

Compared with type *B*, our adopted type *A* achieves the same PSNR value, but on SSIM, it is 0.0008 higher than it, and the parameters are 38K less, which may be related to the fact that we constructed the same channel feature mapping relationship using the weight-sharing convolution layer. Compared with type *C*, type *A* is higher than it by 0.001 on SSIM, which also proves that the weight-sharing auxiliary path can effectively enhance the channel characteristics. In contrast, compared with type *D*, type *A* is 0.04 dB higher in PSNR and 0.0012 higher in SSIM, which shows that type A contributes more to the network performance than type *D* under the same number of parameters.

*To verify the effectiveness of the WSILB design*: we replace the WSILB in PMDN with SE (squeeze-and-excitation), CA (channel attention), and CCA (contrast-aware channel attention), respectively, while the PMDN without attention blocks is used as the baseline, and experimental results are shown in Table 2.

It can be seen clearly from Table 2 that the attention mechanism can effectively improve the performance of the network. Obviously, our PMDN-WSILB is 0.09 dB higher than the baseline on PSNR and 0.001 higher than the baseline on SSIM. Meanwhile, PMDN-WSILB is higher than PMDN-SE and PMDN-CA in two objective indexes. Compared with PMDN-CCA, PMDN-WSILB is 0.02 dB higher on PSNR and 0.0005 higher on SSM. It can be seen that the auxiliary branch in WSILB enhances the channel characteristics and enables WSILB to focus more accurately on information in important channels. Compared with the channel compression and recovery modes used in other attention blocks, WSILB we designed directly uses 1 × 1 convolution layers to model the interdependence between channels in an uncompressed manner, effectively reducing the problem of channel information loss due to channel compression. Although the number of parameters in WSILB is slightly higher than that of other attention blocks, WSILB achieves a good improvement in PSNR and SSIM.

*Verify the effectiveness of DCRB*: we use residual block (RB) composed of two convolution layers and residual attention block (RAB) with WSILB instead of the DCRB in PMDB for experiments, respectively, and the experimental results are shown in Table 3.

Compared with PMDB-RB and PMDB-RAB, our designed PMDB-DCRB achieves the best results in PSNR and SSIM, and the parameters are 113K and 146K less, respectively. DCRB adaptively calibrates the channel feature response and retains the underlying information through another branch, which effectively makes up for the loss of some key information caused by the attention mechanism.

*Verify the effectiveness of the stepwise processing and attention mechanism introduced into the reconstruction process*: to demonstrate that the introduction of the attention mechanism and the stepwise up-sampling strategy in the reconstruction process has a good enhancement effect on the network, we conducted experiments to verify this. The experimental results are shown in Table 4, where U-WSILB-×4 refers to the reconstruction process with WSILB and direct ×4 up-sampling, U-×2-×2^Weightsharing^ means that there is no WSILB in the reconstruction process, the ×4 reconstruction task is divided into two cascaded ×2 reconstruction tasks, and the two reconstruction blocks use the weight-sharing strategy.

Compared with the reconstruction process without attention mechanism, U-WSILB-×4 is 0.03 dB higher than U-×4 on PSNR. Similarly, U-WSILB-×2-×2^Weightsharing^ is 0.02 dB higher than U-×2-×2^Weightsharing^. U-WSILB-×2-×2^Weightsharing^ is 0.0007 higher than U-×2-×2^Weightsharing^ on SSIM, and this effectively proves that introducing WSILB in the reconstruction process can well improve the reconstruction performance of the network.

This shows the effectiveness of the step-by-step strategy in the reconstruction process, and the experimental results are shown in Table 4. Compared with single-step processing, the 0.06 dB of U-×2-×2^Weightsharing^ is higher than that of U-×4 on PSNR, and the 0.05 dB of U-WSILB-×2-×2^Weightsharing^ is higher than that of U-WSILB-×4. On SSIM, U-WSILB-×2-×2^Weightsharing^ is 0.0009 higher than U-WSILB-×4. Obviously, the step-by-step up-sampling processing strategy can ensure that there is enough high-frequency information available for each step of the reconstruction task, thus improving the performance of the network.

To further mitigate the network parameters, we used the weight-sharing strategy for the reconstructed blocks in the reconstruction process. As can be seen from Table 4, U-WSILB-×2-×2^Weightsharing^ is 0.04 dB higher than U-WSILB-×2-×2^Noweight-sharing^ on PSNR and 0.001 higher on SSIM, while the number of parameters is 41 K less.

### 4.3. Compared with Other Excellent Lightweight SR Algorithms

In this paper, the LR images generated by the widely used BI degradation model are used to evaluate the ×2, ×3, and ×4 reconstruction tasks. The proposed PMDN is compared with other reconstruction algorithms, including SRCNN [13], HDRN [16], VDSR [20], MemNet [22], CARN [38], SRMDNF [39], IDN [24], DNCL [40], FilterNet [41], MRFN [42], CFSRCNN [43], LAPAR-B [44], MADNet-LF [45], SMSR [46], ECBSR [47], FDIWN-M [48], and SCFFN [49]. The experimental results are shown in Table 5.

From the experimental data in Table 5, we can see that our PMDN achieves relatively good reconstruction results on the ×2 and ×3 SR tasks compared to some other advanced SR algorithms. For the ×4 SR task, PMDN obtains a good PSNR on Set5, which is 0.003 higher than LAPAR-B and 0.002 higher than SMSR on SSIM. On the B100 data sets, PMDN achieves 0.06 dB higher than ECBSR on PSNR and 0.11 dB higher than MRFN. For Urban100 test set containing rich edge texture content, PMDN outperforms ECBSR by 0.17 dB on PSNR and exceeds ECBSR by 0.007 on SSIM. In short, our PMDN learns the characteristics of each stage feature from coarse to fine by stepwise distillation, allowing the network to learn powerful feature representations effectively, thus showing some advantages in quantitative comparison of reconstruction results.

In addition to the objective metrics comparison with each algorithm, we also performed a visual comparison of the reconstruction results under ×4 reconstruction task, as shown in Figure 5, because the ×4 reconstruction task is a better test of the network's ability to extract and utilize the a priori information. Compared with other algorithms, our PMDN generates relatively clear and reconstructed images containing more edge details on Set5. For Urban-HR-img72, the image generated by VDSR appears severely blurred, while PMDN recovers more building lines with well-defined edge contours compared to IDN, MRFN, and SMSR. For Urban-HR-92, the images generated by other algorithms show severe blurring and line distortion, while our PMDN accurately reconstructs the edges of the building lines and achieves better recovery results.

In addition, in order to compare the performance of each algorithm more comprehensively, we visualize the corresponding relationships between PSNR and the number of parameters and computational complexity of some advanced algorithms under the ×4 reconstruction task as shown in Figures 6 and 7. Compared with some other advanced SR algorithms, the PMDN in this paper achieves a good balance between the number of parameters and performance and shows some competitive advantages, and this makes it possible to apply it to small devices with limited storage. In addition, PMDN achieves a good reconstruction result with low amount of computation, which shows a good balance between performance and computational complexity in Figure 7. In short, our PMDN achieves a good balance between performance, number of parameters, and computational complexity so that our algorithm can be applied to mobile devices with limited memory and computation.

## 5. Conclusions

In this paper, we propose a lightweight and effective progressive multistage distillation network, which abandons the previous crude distillation approach of distilling a small number of features from a large number of input features but adopts a progressive multistage distillation from coarse to fine distillation approach so that the important features of each stage can play its due role. In addition, in order to fully exploit the potential of the network, we design a weight-sharing information lossless attention block, which enhances the channel characteristics through weight-sharing auxiliary branches and then models the relationship between channels without compression by means of convolution layers, avoiding the problem of channel information loss due to channel compression and allowing the network to more accurately distinguish different types of information contained in the channels. Finally, we also introduce the attention mechanism into the reconstruction process and adopt a stepwise up-sampling strategy to enhance the network's attention to high-frequency information, while further employing a weight-sharing strategy to reduce the number of network parameters. Extensive experimental results show that our PMDN shows some advantages in terms of reconstruction results and achieves a good balance between the performance, number of parameters, and computational complexity of the network, allowing our algorithm to be easily applied to small removable devices with limited storage and computational capacity. In addition, the performance of our algorithm needs to be further improved under the condition that device storage and computational capacity are further limited. In the future, we will address these issues and hope to develop lightweight and low-complexity reconstruction algorithms with good results.

## Figures and Tables

**Figure 1:** Overall block diagram of the progressive multistage distillation network. (PMDB stands for progressive multistage distillation block, NNIA stands for nearest neighbor interpolation algorithm, WSILB stands for weight-sharing information lossless attention block, and U-WSILB denotes the reconstruction block containing WSILB).

**Figure 2:** Weight-sharing information lossless attention block (64 refers to 64 channels).

**Figure 3:** (a) Progressive multistage distillation block (PMDB) and (b) dual branch information calibration reservation block (DCRB).

**Figure 4:** Four types of attention blocks.

**Figure 5:** Visual comparison of reconstruction results.

**Figure 6:** Correspondence between PSNR and parameters of each algorithm on the Set5 test set (2022-SCFFN refers to the SCFFN algorithm that appeared in 2022).

**Figure 7:** Correspondence between PSNR and computational complexity of each algorithm.

**Table 1:** Performance comparison between four types of attention blocks.

Attention type	*A*	*B*	*C*	*D*
PSNR(Set5)	32.19	32.19	32.19	32.15
SSIM(Set5)	0.8944	0.8936	0.8934	0.8932
Parameters	781K	819 K	781K	781 K

**Table 2:** Performance comparison for verifying the effectiveness of WSILB.

Attention type	PMDN-No	PMDN-SE	PMDN-CA	PMDN-CCA	PMDN-WSILB
PSNR (Set5)	32.10	32.18	32.13	32.17	32.19
SSIM (Set5)	0.8934	0.8934	0.8929	0.8939	0.8944
Parameters	744K	753 K	753K	754 K	781K

**Table 3:** Performance comparison for verifying the validity of DCRB.

Block type	PMDB-RB	PMDB-RAB	PMDB-DCRB
PSNR (Set5)	32.16	32.18	32.19
SSIM (Set5)	0.8937	0.8936	0.8944
Parameters	894K	927 K	781K

**Table 4:** Performance comparison for verifying the effectiveness of the attention mechanism and distributed processing in the reconstruction phase.

Up-pattern	U-×4	U-WSILB-×4	U-×2-×2^Weightsharing^	U-WSILB-×2-×2^Weightsharing^	U-WSILB-×2-×2^NoWeightsharing^
PSNR (Set5)	32.11	32.14	32.17	32.19	32.15
SSIM (Set5)	0.8929	0.8935	0.8937	0.8944	0.8934
Parameters	777K	781 K	777K	781 K	822K

**Table 5:** Comparison of reconstruction results among algorithms under ×2, ×3, and ×4 reconstruction.

Scale	Method	Set5		Set14		B100		Urban100	
		PSNR	SSIM	PSNR	SSIM	PSNR	SSIM	PSNR	SSIM
*Comparison of ×2 reconstruction results*									
×2	SRCNN	36.66	0.954	32.42	0.906	31.36	0.888	29.50	0.895
	VDSR	37.53	0.959	33.03	0.912	31.90	0.896	30.76	0.914
	MemNet	37.78	0.960	33.28	0.914	32.08	0.898	31.31	0.919
	CARN	37.76	0.959	33.52	0.917	32.09	0.898	31.92	0.926
	SRMDNF	37.79	0.960	33.32	0.915	32.05	0.898	31.33	0.920
	IDN	37.83	0.960	33.30	0.915	32.08	0.898	31.27	0.920
	DNCL	37.65	0.960	33.18	0.914	31.97	0.897	30.89	0.916
	FilterNet	37.86	0.961	33.34	0.915	32.09	0.899	31.24	0.920
	MRFN	37.98	0.961	33.41	0.916	32.14	0.899	31.45	0.922
	CFSRCNN	37.79	0.959	33.51	0.916	32.11	0.898	32.07	0.927
	LAPAR-B	37.87	0.960	33.39	0.916	32.10	0.898	31.62	0.924
	MADNet-L_F_	37.85	0.960	33.39	0.916	32.05	0.898	31.59	0.923
	SMSR	38.00	0.960	33.64	0.918	32.17	0.899	32.19	0.928
	ECBSR	37.90	0.962	33.34	0.918	32.10	0.902	31.71	0.925
	HDRN	37.75	0.959	33.49	0.915	32.03	0.898	31.87	0.925
	SCFFN	38.01	0.960	33.52	0.917	32.12	0.899	31.39	0.926
	PMDN	37.95	0.960	33.58	0.918	32.16	0.899	32.10	0.927

*Comparison of ×3 reconstruction results*									
×3	SRCNN	32.75	0.909	29.28	0.821	28.41	0.786	26.24	0.799
	VDSR	33.66	0.921	29.77	0.831	28.82	0.798	27.14	0.828
	MemNet	34.09	0.925	30.00	0.835	28.96	0.800	27.56	0.838
	CARN	34.29	0.925	30.29	0.841	29.06	0.803	28.06	0.849
	SRMDNF	34.12	0.925	30.04	0.837	28.97	0.803	27.57	0.840
	IDN	34.11	0.925	29.99	0.835	28.95	0.801	27.42	0.836
	DNCL	33.95	0.923	29.93	0.834	28.91	0.799	27.27	0.833
	FilterNet	34.08	0.925	30.03	0.837	28.95	0.803	27.55	0.838
	MRFN	34.21	0.927	30.03	0.836	28.99	0.803	27.53	0.839
	CFSRCNN	34.24	0.926	30.27	0.841	29.03	0.803	28.04	0.850
	LAPAR-B	34.20	0.926	30.17	0.839	29.03	0.803	27.85	0.846
	MADNet-L_F_	34.14	0.925	30.20	0.839	28.98	0.802	27.78	0.844
	SMSR	34.40	0.927	30.33	0.841	29.10	0.805	28.25	0.854
	HDRN	34.24	0.924	30.23	0.840	28.96	0.804	27.93	0.849
	SCFFN	34.29	0.926	30.27	0.841	29.04	0.803	27.98	0.848
	PMDN	34.36	0.926	30.29	0.840	29.07	0.804	28.15	0.852

*Comparison of ×4 reconstruction result*									
×4	SRCNN	30.48	0.863	27.49	0.750	26.90	0.710	24.52	0.722
	VDSR	31.35	0.884	28.01	0.767	27.29	0.725	25.18	0.752
	MemNet	31.74	0.889	28.26	0.772	27.40	0.728	25.50	0.763
	CARN	32.13	0.894	28.60	0.781	27.58	0.735	26.07	0.784
	SRMDNF	31.96	0.893	28.35	0.777	27.49	0.734	25.68	0.773
	IDN	31.82	0.890	28.25	0.773	27.41	0.730	25.41	0.763
	DNCL	31.66	0.887	28.23	0.772	27.39	0.728	25.36	0.761
	FilterNet	31.74	0.890	28.27	0.773	27.39	0.729	25.53	0.768
	MRFN	31.90	0.892	28.31	0.775	27.43	0.731	25.46	0.765
	CFSRCNN	32.06	0.892	28.57	0.780	27.53	0.733	26.03	0.782
	MADNet-L_F_	32.01	0.892	28.45	0.778	27.47	0.733	25.77	0.775
	LAPAR-B	31.94	0.892	28.46	0.778	27.52	0.734	25.85	0.777
	SMSR	32.12	0.893	28.55	0.781	27.55	0.735	26.11	0.787
	FDIWN-M	32.17	0.894	28.55	0.781	27.58	0.736	26.02	0.784
	ECBSR	31.92	0.895	28.34	0.782	27.48	0.739	25.81	0.777
	HDRN	32.23	0.896	28.58	0.781	27.53	0.737	26.09	0.787
	SCFFN	32.18	0.895	28.56	0.781	27.54	0.735	26.01	0.783
	PMDN	32.27	0.895	28.58	0.781	27.54	0.735	25.98	0.784

## Data Availability

Publicly available data sets were analyzed in this study. Our training set DIV2k and Flickr2K data sets can be obtained online (DIV2K data sets: https://data.vision.ee.ethz.ch/cvl/DIV2K/; Flickr2K data sets: http://cv.snu.ac.kr/research/EDSR/Flickr2K.tar). Set5, Set14, B100, and Urban 100 can be obtained online (https://arxiv.org/abs/1909.11856). In order to facilitate the reproduction of the experimental results, we specially attach the code link: https://github.com/Cai631/PMDN.
